The article "Optimization of diosgenin extraction from Dioscorea deltoidea tubers using response surface methodology and artificial neural network modelling" was retracted in 2023. Reasons: errors in the images; duplicated images; overlap with earlier publications; a conflict of interest.

# Optimization of diosgenin extraction from *Dioscorea deltoidea* tubers using response surface methodology and artificial neural network modelling

**DOI:** 10.1371/journal.pone.0253617

**Published:** 2021-07-21

**Authors:** Romaan Nazir, Devendra Kumar Pandey, Babita Pandey, Vijay Kumar, Padmanabh Dwivedi, Aditya Khampariya, Abhijit Dey, Tabarak Malik

**Affiliations:** 1 Department of Biotechnology, Lovely Faculty of Technology and Sciences, Lovely Professional University, Phagwara, Punjab, India; 2 Department of Computer Science and Information Technology, Babasaheb Bhimrao Ambedkar University, Lucknow, Uttar Pradesh, India; 3 Department of Plant Physiology, Banaras Hindu University, Varanasi, Uttar Pradesh, India; 4 School of Computer Science and Engineering, Lovely Professional University, Phagwara, Punjab, India; 5 Department of Life Sciences, Presidency University, Kolkata, India; 6 Department of Biochemistry, College of Medicine and Health Sciences, University of Gondar, Gondar, Ethiopia; Ton Duc Thang University, VIET NAM

## Abstract

**Introduction:**

*Dioscorea deltoidea* var. *deltoidea* (Dioscoreaceae) is a valuable endangered plant of great medicinal and economic importance due to the presence of the bioactive compound diosgenin. In the present study, response surface methodology (RSM) and artificial neural network (ANN) modelling have been implemented to evaluate the diosgenin content from *D*. *deltoidea*. In addition, different extraction parameters have been also optimized and developed.

**Materials and methods:**

Firstly, Plackett-Burman design (PBD) was applied for screening the significant variables among the selected extraction parameters i.e. solvent composition, solid: solvent ratio, particle size, time, temperature, pH and extraction cycles on diosgenin yield. Among seven tested parameters only four parameters (particle size, solid: solvent ratio, time and temperature) were found to exert significant effect on the diosgenin extraction. Moreover, Box-Behnken design (BBD) was employed to optimize the significant extraction parameters for maximum diosgenin yield.

**Results:**

The most suitable condition for diosgenin extraction was found to be solid: solvent ratio (1:45), particle size (1.25 mm), time (45 min) and temperature (45°C). The maximum experimental yield of diosgenin (1.204% dry weight) was observed close to the predicted value (1.202% dry weight) on the basis of the chosen optimal extraction factors. The developed mathematical model fitted well with experimental data for diosgenin extraction.

**Conclusions:**

Experimental validation revealed that a well trained ANN model has superior performance compared to a RSM model.

The article "Optimization of diosgenin extraction from Dioscorea deltoidea tubers using response surface methodology and artificial neural network modelling" was retracted in 2023. Reasons: errors in the images; duplicated images; overlap with earlier publications; a conflict of interest.

## 1. Introduction

The tubers of several species of the genus Dioscorea (Family: Dioscoreaceae) contain steroidal saponins and sapogenins (diosgenin), which is the preliminary material of industrial interest in the synthesis of many steroidal drugs which are on the market as antitumor, anti-inflammatory, anticancer, androgenic, estrogenic, and contraceptive drugs [1]. One of the important species is *D*. *deltoidea var*. *deltoidea* is a climbing herb having rhizomatous rootstock. It is found in the tropical and sub-tropical areas of the world, mostly present in Pakistan, Bhutan, Vietnam, India, Nepal and China. In India, it is mainly distributed in Assam to Kashmir at altitudes of 550–3100 m [2]. In Himalayan regions this plant grows in Assam, Sikkim, Uttarakhand, Jammu and Kashmir, Meghalaya and Arunanchal Pradesh [3]. *D*. *deltoidea* contains a variety of bioactive compounds such as stigmasterol, diosgenin and other sapogenins [1], among which, diosgenin has been considered as most important phytochemical compound and foremost source for the endorsement of *D*. *deltoidea*. Diosgenin is a steroidal sapogenin used as a precursor of sex hormones (progesterone), corticosteroids (corticosone) and contraceptives [4, 5]. This compound is also used as a supplement by body builders to build muscle mass and to increase testosterone level [6]. Traditionally, it is used as an anti-diabetic, anti-hypertriacylglycerolimia, anti-hypercholesterolemia, anti-hyperglycemic and anti-leukemia agent [7].

Currently, its demand is increasing day by day in pharmaceutical industries due to its immense therapeutic activities such as anti-cancer [8, 9], anti-diabetic [10, 11], anti-fungal [12], anti-viral [13], anti-microbial [14], anti-tumour [15], anti-oxidant [16, 17], anti-coagulant and anti-thrombosis [18, 19] activities. In addition, it also shows effects on skin aging [20, 21], menopausal symptoms [22, 23], CNS [24], lipid system [25] and blood pressure.

Diosgenin is a commercially important bioactive compound, therefore optimization of isolation and purification of this compound by different extraction procedures is crucial. Many other factors such as extraction time, method, cycle, temperature, solvent type, solid: solvent ratio, particle size, and pH are stated to influence the total diosgenin content [26–30]. Different conventional extraction methods such as soxhlet [31, 32], heat reflux [33] ultrasonic assisted extraction (UAE) and liquid-liquid extraction (LLE) [34] have been used for the extraction of diosgenin. Specialized and reproducible extraction methods for the isolation of valuable bioactive compounds from several plant species including Himalayan plants is still lacking [26, 35]

In recent years researchers were investigating specific extraction condition for the optimization of high yield of bioactive compounds from different medicinal plant species. However, considering a one-factor-at-a-time is time consuming, expensive and less effective and lacks interactive effect of factors influencing extraction. On the other hand, response surface methodology (RSM) is a statistical techniques for designing experiments, building models and considered as highly effective tool for optimization of various factors for the better yield [36, 37]. RSM is broadly employed for enhancing the extraction of vitamin E, phenolic compounds, polysaccharides, polyphenolics, triterpenoids, anthocyanins, xanthonoids and protein from various plant resources [37–45]. It is also used to achieve maximum Remazol brilliant blue R (RBBR) dye decolourization and chemical oxygen demand (COD) reduction, to optimize the key parameters for methylene blue dye adsorption, reactive orange 16 (RO16) dye adsorption and adsorptive properties of chitosan-tripolyphosphate/ fly ash(CS-TPP/FA) for removal of reactive red (RR120) dye from the aqueous environment [46–49]. Whereas, Artificial Neural Network (ANN) is a data processing approach based on the non-linear weighted sum statistical data modelling tools [46, 47]. ANN is inspired of biological neuron network that determines an intricate association between the responses and predicted variables [48]. This modelling technique allows computing, learning, and memorizing as similar as human brains [49]. ANN as compared to RSM is more precise technique of interpolation, prediction, and validation [46]. The present research focuses on the optimization of extraction parameters on diosgenin from *D*. *deltoidea*. Consecutively, the results predicted by RSM and ANN were compared with the experimental value for their accuracy and generalization capability. To the best of our knowledge no reports have been published so far on heat reflux extraction of diosgenin from *D*. *deltoidea* and comparative study between RSM and ANN on diosgenin. The present investigation was undertaken with the objective to screen the significant extraction parameters by applying PBD, to maximize the yield of diosgenin from tubers of *D*. *deltoidea*, RSM with BBD as a powerful optimization approach was applied in order to optimize the extraction process parameters such as solid: solvent ratio, particle size, temperature and time. Furthermore, ANN model were applied, and compared with RSM model.

The article "Optimization of diosgenin extraction from Dioscorea deltoidea tubers using response surface methodology and artificial neural network modelling" was retracted in 2023. Reasons: errors in the images; duplicated images; overlap with earlier publications; a conflict of interest.

## 2. Materials and methods

### 2.1 Chemicals and plant material

*D*. *deltoidea* plant with tuber was collected from a local nursery from Chakrata district, Uttarakhand, India. The plant was identified by the taxonomist and voucher specimen (15062018) was kept in School of Bioengineering and Biosciences, Lovely Professional University. The freshly collected tubers were rinsed using water followed by drying in shade at room temperature. Dried tubers were ground into fine powder in electric grinder. The powdered samples were sieved into three different homogeneous particle sizes (0.50 mm; mesh size 35, 1.25 mm; mesh size 16 and 2.00 mm; mesh size 10) and stored in airtight glass bottles (51, 52).

Methanol, chloroform (HPLC grade), ethanol was purchased from Thomas Baker (Mumbai, India). Ultra-pure water was obtained from a Milli Q PLUS purification system (Millipore, USA). The standard diosgenin (Fig 1) were procured from Sigma-Aldrich, USA. All chemicals used in the assays were of analytical grade. HPTLC plates (0.25mm): pre-coated silica gel 60 F254 were procured from Merck, Darmstadt, Germany. Rotary evaporator (SJW, Ambala), centrifuge machine (REMI, Ambala), and mixer grinder (Philips HL1606/03) were used in conducting the extraction and sample preparation.

**Fig 1:** Chemical structure of diosgenin.

### 2.2 Extraction of diosgenin

The heat reflux extraction (HRE) was performed in a temperature controlled heater using round bottom flask equipped with condenser to avoid solvent evaporation. The anhydrous dry powder samples (1.0 g) were extracted using different volumes of solvent (ethanol: water mixtures) according to experimental design (PBD and BBD). To evaluate the influence of solid: solvent extraction on the diosgenin yield, tests were carried out via different extraction variables *viz*., solvent composition (X_1_:Ethanol-water), solid-to-solvent ratio (X_2_:30–60 ml g^–1^), particle size (X_3_: 0.5–2.05), extraction time (X_4_:30–60 min), temperature (X_5_:30–60°C), pH (X_6_:5–9), and extraction cycles (X_7_:1–3). After extraction, samples were filtered, concentrated to dryness in a rotary evaporator at 40°C. 20 ml of HCL (10%) was added to the dried residue and heated to hydrolyse for 60 min in water bath at 98°C. After cooling, two times 15 ml chloroform were used for washing and collective mixture was extracted and segregated, the chloroform layer i.e. lower layer was collected and further 20 ml chloroform was used to extract upper layer. All the collected chloroform layers were combined and concentrated to dryness. An appropriate amount of methanol was added to the residue and the final concentration was filtered through 0.45μm polypropylene membrane filter before high performance thin layer chromatography (HPTLC) analysis.

### 2.3 HPTLC method for assessment of diosgenin content

Estimation of diosgenin was carried out by using HPTLC analysis comprised of Linomat–5 applicator CAMAG (Switzerland) fitted with 100μl syringe and TLC scanner-3 CAMAG (Switzerland) run by win CATS software (version: 1.4.6.2002) for better data collection and documentation. The stationary phase used was 20 × 10 cm precoated silica gel 60 F_254_ TLC plates. The samples were patched in form of A 6mm-wide bands to the plates. The mobile phase used was toluene: chloroform: acetone (2:8:2) saturated in CAMAG twin trough chamber. Post-derivatization of plates was done by anisaldehyde reagent (1 ml anisaldehyde, 20 ml glacial acetic acid, 170 ml methanol and 10 ml conc. sulphuric acid), heated for 5 min at 100°C.

The article "Optimization of diosgenin extraction from Dioscorea deltoidea tubers using response surface methodology and artificial neural network modelling" was retracted in 2023. Reasons: errors in the images; duplicated images; overlap with earlier publications; a conflict of interest.

### 2.4 Preparation of standard calibration curve of diosgenin

For preparation of calibration curves of diosgenin (0.1 mg. ml^-1^ in methanol), different concentrations of working standard solution [2 μl (200 ng), 4 μl (400 ng), 6 μl (600 ng), 8 μl (800 ng), and 10 μl (1000 ng)] were applied to obtain linearity range of 200–1000 ng/spot. Densitometric scanning was performed at λ = 433 nm.

### 2.5 Validation of method

Method validation was performed according to the guidelines of International Conference on Harmonisation (ICH) on the parameters such as linearity, limit of sensitivity, specificity, precision, accuracy, recovery, and robustness presented in Table 1 [50].

**Table 1:** Method validation for diosgenin quantification.

S.No	Parameters	Value
**1**	Linearity range (ng/spot;*n* = 12^a^)	200–1000
**2**	Correlation coefficient (r^2^)	0.993
**3**	Regression equation	Y = 15.25X + 26424
**4**	Calculated SD value	0.32
**5**	^b^Limit of detection (LOD) (ng) [3×SD/S]	20
**6**	^b^Limit of quantification (LOQ) (ng) [10×SD/S]	60
**7**	R_f_	0.78
**Precision and accuracy**		
**8**	Intra-day^c^ RSD (%), n = 5	1.34
**9**	Inter-day RSD (%), n = 5	1.56
**Recovery**		
**10**	Amount of standard in plant samples (μg mg^−1^) containing highest bioactive compounds	12.04
**11**	Amount of standards added in plant samples (μg mg^−1^)	6, 12, 18
**12**	Amount of standard found (μg mg^−1^)	18.15, 23.98, 29.98
**13**	Recovery (%)	100.6, 99.75, 99.80
**14**	Mean Recovery (%)	100.05

^a^ Five concentration levels in triplicate.

^b^ SD is the standard deviation of the blank response and S is the slope of the calibration plot.

^c^RSD is Relative standard deviation; RSD = 100S / x−; S: standard deviation; x: mean.

### 2.6 Modelling and optimization studies

Investigation was performed via two phases: Plackett-Burmandesign (PBD) was employed to analyse the significant independent parameters and Box-Behnken design (BBD) applied to check the optimal level and probable collaborations among significant parameters. Experimental design was set up in Minitab software. Furthermore, Design Expert software, version 12 was used to generate 3 D surface plot.

The article "Optimization of diosgenin extraction from Dioscorea deltoidea tubers using response surface methodology and artificial neural network modelling" was retracted in 2023. Reasons: errors in the images; duplicated images; overlap with earlier publications; a conflict of interest.

#### 2.6.1 Plackett–Burman design (PBD)

PBD was employed for the optimization of diosgenin to estimate the significant parameters. This model depends on first-order model:

Y=β0+∑βiXi (1)

Where expected target function is denoted by *Y*, scaling constant is *β*_*0*_ and a regression coefficient is *β*_*i*._ The influence of independent variables *viz*., time, pH, solid: solvent ratio, solvent composition, temperature, extraction steps as well as the particle size on diosgenin was tested. Test was directed at two levels in which (+) implies greatest esteem and (-) implies least esteem (portrayed in Table 2). All factors said above were tried in triplicates by directing 12 tests (plot portrayed in Table 3). Regression analyses at 5% (*p < 0*.*05*) have been used to test the significant factors, as appeared in Table 4.

**Table 2:** Different extraction parameters used for diosgenin extraction from *D*. *deltoidei*.

Variable code	Variables	High level(+)	Low level(-)
**X**_**1**_	Solvent Composition (Ethanol and water)	100	0
**X**_**2**_	Solid: solvent ratio(g/ml)	1:60	1:30
**X**_**3**_	Particle size (mm)	2.00	0.5
**X**_**4**_	Time (min)	60	30
**X**_**5**_	Temperature (°C)	60	30
**X**_**6**_	pH	9	5
**X**_**7**_	Cycles/steps	3	1

**Table 3:** Diosgenin content from *D*. *deltoidea* tuber using different levels of extraction variables of Plackett-Burman design criteria.

Runs	X_1_	X_2_	X_3_	X_4_	X_5_	X_6_	X_7_	(%)Diosgenin
1	1	-1	-1	1	-1	-1	1	1.016
2	-1	-1	1	1	1	-1	-1	0.906
3	1	1	-1	-1	1	-1	-1	0.907
4	1	-1	1	1	-1	1	-1	0.909
5	-1	1	1	1	1	-1	1	0.477
6	1	1	-1	1	1	1	-1	0.964
7	1	-1	1	-1	1	1	1	0.953
8	1	1	1	-1	-1	-1	1	0.957
9	-1	1	1	-1	-1	1	-1	0.637
10	-1	1	-1	1	-1	1	1	0.464
11	-1	-1	-1	-1	1	1	1	0.758
12	-1	-1	-1	-1	-1	-1	-1	0.393

**Table 4:** Regression analysis for prediction of significant extraction parameters by PBD criterion.

Term	Effect	Coefficient	SE coefficient	*T*	*P*
**Constant**		0.782	0.022	34.50	0.000
**Particle size**	0.141	0.070	0.022	3.11	0.036
**Solid: Solvent ratio**	0.175	0.087	0.022	3.86	0.018
**Time**	0.403	0.201	0.022	8.90	0.001
**Temperature**	0.123	0.061	0.022	2.72	0.049
**Solvent composition**	-0.078	-0.039	0.022	-1.73	0.158
**pH**	-0.004	-0.002	0.022	-0.10	0.928
**Extraction cycles**	0.026	0.013	0.022	0.59	0.588

#### 2.6.2 Box-Behnken design (BBD)

BBD is somewhat a spherical, revolving quadratic and independent model with no fixed fractional factorial points wherever the combinations are at the midpoints of the edges and at the centre of the variable space [51]. In this study, BBD was utilized to examine the combined impact of four independent variables i.e., solid: solvent ratio, time, temperature as well as size of particle on diosgenin extraction, which was previously selected by PBD. In this model, three variable levels i.e., low, middle and high (-1, 0, +1) were tested, (as shown in Table 5). According to the equation given below, the coding of variables was done [52]:

$$\begin{array}{ll} \text{xi}=\text{Xi}–\text{X}0/\Delta \text{Xi} & \text{i}=1,2,3\ldots ,\text{k} \end{array}$$ (2)

Where x_i_ represents independent variable of coded value; X_i_ represents independent variable of actual value; X_0_ is the independent variable of the actual value at the centre point; and ΔX_i_ is the independent variable of the step change value. In BBD, a total number of 27 runs were accomplished and the results are recorded in Table 6. All experiments were executed in triplicates and the averages of diosgenin content were taken as response.

The article "Optimization of diosgenin extraction from Dioscorea deltoidea tubers using response surface methodology and artificial neural network modelling" was retracted in 2023. Reasons: errors in the images; duplicated images; overlap with earlier publications; a conflict of interest.

**Table 5:** Actual and coded treatment variables for optimization of diosgenin extraction from *D*. *deltoidea* using BBD.

Variables	Coded levels				
		Codes	+ 1	0	-1
**Solid: Solvent ratio (g/ml)**	X_2_	A	60	45	30
**Particle size (mm)**	X_3_	B	2.00	1.25	0.5
**Extraction time (min)**	X_4_	C	60	45	30
**Temperature (°C)**	X_5_	D	60	45	30

**Table 6:** Experimental and predicted value of BBD design with four different extraction variables: Solid: Solvent ratio(X_2_), particle size (X_3_), time (X_4_) and temperature(X_5_).

Run order	Factors				Diosgenin (% dry weight)		
	Solid: solvent ratio (X_2_)	Particle size (X_3_)	Time (X_4_)	Temperature(X_5_)	Experimental	RSM Predicted	ANN
**1**	30	0.50	45	45	1.128	1.151	1.129
**2**	60	0.50	45	45	1.151	1.150	1.153
**3**	30	2.00	45	45	1.151	1.134	1.152
**4**	60	2.00	45	45	1.135	1.126	1.137
**5**	45	1.25	30	30	1.127	1.128	1.128
**6**	45	1.25	60	30	1.129	1.146	1.132
**7**	45	1.25	30	60	1.147	1.151	1.147
**8**	45	1.25	60	60	1.152	1.156	1.155
**9**	30	1.25	45	30	1.156	1.116	1.155
**10**	60	1.25	45	30	1.117	1.133	1.118
**11**	30	1.25	45	60	1.134	1.181	1.133
**12**	60	1.25	45	60	1.182	1.125	1.183
**13**	45	0.50	30	45	1.126	1.135	1.128
**14**	45	2.00	30	45	1.135	1.135	1.134
**15**	45	0.50	60	45	1.137	1.131	1.137
**16**	45	2.00	60	45	1.132	1.119	1.138
**17**	30	1.25	30	45	1.119	1.137	1.119
**18**	60	1.25	30	45	1.137	1.136	1.137
**19**	30	1.25	60	45	1.135	1.126	1.135
**20**	60	1.25	60	45	1.125	1.144	1.125
**21**	45	0.50	45	30	1.144	1.133	1.144
**22**	45	2.00	45	30	1.133	1.151	1.134
**23**	45	0.50	45	60	1.150	1.169	1.15
**24**	45	2.00	45	60	1.169	1.204	1.168
**25**	45	1.25	45	45	1.202	1.204	1.191
**26**	45	1.25	45	45	1.201	1.204	1.192
**27**	45	1.25	45	45	1.211	1.151	1.192

To compare the relationship between independent variables and diosgenin content a second-order polynomial equation was applied for the prediction of optimal point. The equation for four variables is given below:

$$\begin{array}{c} Y=\beta 0+\beta 2X2+\beta 3X3+\beta 4X4+\beta 5X5+\beta 22X22+\beta 33X32+\beta 44X42+\beta 55X52\\ +\beta 23X2X3+\beta 24X2X4+\beta 25X2X5+\beta 34X3X4+\beta 35X3X5 \end{array}$$ (3)

Where Y represents predicted response; *β*_*0*_ shows modal constant; X_2_, X_3_, X_4_ andX_5_ are significant factors; *β*_*2*,_ *β*_*3*,_ *β*_*4 and*_ *β*_*5*_ are linear coefficients; *β*_*22*,_ *β*_*33*,_ *β*_*44*_ and *β*_*55*_ are quadratic coefficients and *β*_*23*,_ *β*_*24*,_ *β*_*25*,_ *β*_*34*,_ *β*_*35*,_ *β*_*45*_ are the interactive coefficients. Diosgenin content in *D*. *deltoidea* has been evaluated by the regression coefficient and ANOVA. 3-D surface plots of % diosgenin were prepared for each interactive coefficient by Design Expert 12 software (Fig 4A-4F).

The article "Optimization of diosgenin extraction from Dioscorea deltoidea tubers using response surface methodology and artificial neural network modelling" was retracted in 2023. Reasons: errors in the images; duplicated images; overlap with earlier publications; a conflict of interest.

#### 2.6.3 Artificial Neural Network (ANN) modeling

The functionality of ANN is to alter the given input vectors furnished to model into feature map or output with help of unique rules. In proposed approach multi-layer, perceptron model was utilized by using MATLAB (The Mathworks Inc., 2012a) which comprised of hidden neurons for generation of approximate multi-layer model. The predicted output computation is expressed with help of Eq (4) as:

$$Y=f\left(A_{z}\right)=\overset{m}{\underset{p=1}{\sum }}w_{zp}*x_{p}+\theta_{z}$$ (4)

Here, *Y* represents the output obtained from output layer, *f*(*A*_*z*_) denoted the activation functions which is responsible for non-linear nature of model associated with neuron z. *w*_*zp*_ represents weight connection between neuron z and p. *θ*_*z*_ denotes the input bias and *x*_*p*_ illustrated the inputs given to neuron *p*.

To minimize the error and achieve faster convergence, ANN adopted back propagation algorithm during training phase for model training and convergence without any delay or loss. Due to consideration of appropriate neuron size, the obtained achieved results are sound and accurate without any compromises. The multilayer perceptron model consists of four inputs, one hidden and output layer for prediction. For training and validation analysis, Log Sigmoidal function is used as an activation unit for non-linear output prediction. For synaptic weight adjustment and analysis training data is trained with help of Marquardt algorithm and validation is supported and performed with the help of 5-fold cross validation strategy. Fig 6A depicted the performance data obtained over entire training data and fitted at best epochs for validation data being represented. Similarly, gradient loss and training state achieved over entire ANN training is explained with help of Fig 6.

The article "Optimization of diosgenin extraction from Dioscorea deltoidea tubers using response surface methodology and artificial neural network modelling" was retracted in 2023. Reasons: errors in the images; duplicated images; overlap with earlier publications; a conflict of interest.

In addition, comparison was drawn between two models on the basis of three significant statistical parameters, *viz*. Root mean square error (RMSE), Absolute average deviation (AAD) and regression coefficient (*r*^*2*^).

RMSE and AAD were calculated on the basis of Eqs 5 and 6.


$$\text{RMSE}=\left(\frac{1}{n}\overset{\text{n}}{\underset{\text{i}=1}{\sum }}{\left(Y_{predicted}-Y_{experimental}\right)}^{2}\right)\frac{1}{2}$$ (5)

$$AAD(\%)=\left(\overset{\text{P}}{\underset{\text{i}=1}{\sum }}\left(\left|Y_{i,exp}-Y_{i,cal}\right|/Y_{i,exp}\right)/P\right)\times 100$$ (6)

## 3. Results

In the present study, HPTLC analysis has been implicated for the estimation of diosgenin content in different extracts. HPTLC fingerprinting and chromatogram showed the presence of diosgenin (green colour; R_f_: 0.78) in extracts of *D*. *deltoidea* tubers (Fig 2A & 2B). Table 1 showed the analytical characteristics of the method of validation of diosgenin. The linear regression analysis data for the calibration plots Y = 15.25X + 26424) revealed good linear relationship with R^2^ = 0.993 for diosgenin in terms of peak area with concentration range of 200–1000 ng/spot (Fig 3).

**Fig 2:** **A** HPTLC fingerprinting of BBD samples (1–27) after derivatizing by anisaldehyde regent. **B** Chromatogram I of BBD samples (1–14); Chromatogram II of BBD samples (15–27).

**Fig 3:** Calibration plot for diosgenin.

### 3.1 Screening of significant extraction parameters

PBD was employed for the screening and estimation of the effect of seven different parameters on the diosgenin yield (Table 2). The particular design matrix and resultant % diosgenin yield acquired from *D*. *deltoidea* tubers are displayed in Table 3. Regression analysis was used for the screening of the impact of extraction factors (Table 4). Among seven parameters only for parameters (particle size, solid: solvent ratio, time and temperature) had revealed significant impact on diosgenin extraction as shown by their *P* values (*P*< 0.05) given in Table 4. In this study, according to the PBD, the diosgenin yield has shown deviation up to 0.393–1.01%.

### 3.2 Effect of process variables

Investigational design is comprehensively utilized for knowing the influence of parameters in a procedure to diminish the number of tests, material assets and time. Moreover, the experiment implemented on the outcomes effectively acknowledged, and thus the test errors are reduced. The impacts of variations in the test variables are measured by the statistical procedures and their mutual interactions through the investigational design [53]. In this scheme, four parameters at three level BBD was utilised to optimize and examine the effect of independent variables on diosgenin of *D*. *deltoidea* tubers extract obtained by solid–liquid extraction method (Table 5) and the results along with experimental values and predicted values achieved by model equation were shown in Table 6. The quadratic model impact is statistically significant (0.0001) and R^2^ and adjusted R^2^ values of 0.9967 and 0.982 correspondingly, and lack of fit was not significant (1.0). This predicts the adequacy of the model. The quadratic model is observed to be the most appropriate model for the current extraction process.

The article "Optimization of diosgenin extraction from Dioscorea deltoidea tubers using response surface methodology and artificial neural network modelling" was retracted in 2023. Reasons: errors in the images; duplicated images; overlap with earlier publications; a conflict of interest.

Multiple regression analysis was employed on experimental results, providing second-order polynomial Eq 7

$$\begin{array}{c} \text{Y}=1.2046+0.002{\;\;\text{X}}_{2}+0.00158{\;\text{X}}_{3}+0.00158{\text{X}}_{4}+0.01067{\text{X}}_{5}\;\text{--}0.03321\;{\text{X}}_{2}{}^{2}\;\text{-}\;\text{-}0.03058{\text{X}}_{3}{}^{2}\;\text{-}\;\text{-}0.04183{\text{X}}_{4}{}^{2}\\ \text{--}0.02446{\text{X}}_{5}{}^{2}\;\text{-}\;\text{-}0.00975{\text{X}}_{2}{\text{X}}_{3}\;\text{-}\;0.00700{\;\text{X}}_{2}{\text{X}}_{4}+0.02175\;{\text{X}}_{2}{\text{X}}_{5}\;\text{-}\;\text{-}0.00350{\text{X}}_{3}{\text{X}}_{4}+0.00750{\text{X}}_{3}{\text{X}}_{5} \end{array}$$ (7)

The influence of solid: solvent (X_2_), particle size (X_3_), time (X_4_) and temperature (X_5_) on the extraction of diosgenin were shown in Table 7. Regression coefficients had shown significant positive linear effects of the four variables (X_2_, X_3_, X_4_ and X_5_). Among four parameters, temperature has revealed maximum effect on diosgenin yield, by giving the maximum linear coefficient value (0.01067) followed by solid: solvent ratio (0.002), while time (0.00158) and particle size (0.00158) has equal effect. Regression analysis also indicated high significance (p < 0.0001) of model equation terms: main, squared, and interaction effects of process variables. The smaller the magnitude of the P, the more significant is the corresponding coefficient. Values of P less than 0.05 indicate model terms are significant. The significant linear, (X_2_, X_3_, X_4_ and X_5_), quadratic (X_2_^2^, X_3_^2^, X_4_^2^ and X_5_^2^) and interactive effect i.e particle size and time (X_25_), solid: solvent and particle size (X_23_), solid: solvent and time (X_24_), solid: solvent and temperature (X_25_), particle size and time (X_34_) and particle size and temperature (X_35_) were shown in the model regression Eq (4) except time and temperature (X_45_), which had non-significant effect on diosgenin yield. For all the responses such as solid: solvent ratio (X_2_), particle size (X_3_), time (X_4_) and temperature (X_5_) quadratic effect of variables were seen to be significant.

The article "Optimization of diosgenin extraction from Dioscorea deltoidea tubers using response surface methodology and artificial neural network modelling" was retracted in 2023. Reasons: errors in the images; duplicated images; overlap with earlier publications; a conflict of interest.

**Table 7:** Regression analysis of BBD criterion data for diosgenin extraction from *D*. *deltoidea* tuber.

Model parameters	Regression coefficient	S.E.Cofficient	*T*	*P*
**Constant**	1.204	0.001	861.351	0.000
**Solid:Solvent**	0.002	0.001	2.860	0.014
**Particle size**	0.001	0.001	2.264	0.043
**Time**	0.001	0.001	2.264	0.043
**Temperature**	0.010	0.001	15.254	0.000
**Solid:Solvent**^**2**^	-0.033	0.0010	-31.659	0.000
**Particle size**^**2**^	-0.030	0.0010	-29.157	0.000
**Time**^**2**^	-0.041	0.0010	-39.882	0.000
**Temperature**^**2**^	-0.024	0.001	-23.317	0.000
**Solid:Solvent × Particle size**	-0.009	0.001	-8.050	0.000
**Solid:Solvent × Time**	-0.007	0.001	-5.779	0.000
**Solid:Solvent × Temperature**	0.021	0.001	17.957	0.000
**Particle size ×Time**	-0.003	0.001	-2.890	0.014
**Particle size × Temperature**	0.007	0.001	6.192	0.000
**Time × Temperature**	0.001	0.001	0.619	0.547

R-Sq = 99.67% R-Sq(pred) = 98.20% R-Sq(adj) = 99.28%.

ANOVA analysis specifies the linear, interactive and quadratic relationship among the independent variables on their dependent variables [54]. ANOVA for the extraction of diosgenin attained from this model were shown in Table 8. Model values obtained by the Analysis of variance describe whether this model is fit for the variation found in diosgenin extract. If the significance in F-Test is found at the 5% level (*P*< 0.05), then the model can clearly explain the variations and is fit for the analysis [55–58]. The coefficient of determination (*R*^*2*^) value of 0.996 and an adjusted-*R*^*2*^ value of 0.982 appear close to the unity and indicate a high correlation between the actual and the predicted values [59, 60] and R^2^ value (0.9967) indicates that the model can explain the variation up to 99.67% in the extract of diosgenin. The *P* value (1.0) explains that the applied model is fit and also describes the influence of solid: solvent ratio, particle size, time and temperature on diosgenin from *D*. *deltoidea*.

**Table 8:** Analysis of variance for diosgenin extraction from *D*. *deltoidea* by using BBD criterion.

Source	DF	Seq SS	AdjSS	Adj MS	F	P
**Regression**	14	0.016	0.016	0.001	203.85	0.000
**Linear**	4	0.001	0.001	0.001	62.78	0.000
**Square**	4	0.011	0.011	0.001	533.77	0.000
**Interaction**	6	0.002	0.002	0.001	77.96	0.000
**Residual Error**	12	0.0001	0.001	0.000		
**Lack-of-Fit**	10	0.001	0.001	0.000	0.03	1.000
**Pure Error**	2	0.001	0.001	0.000		
**Total**	26	0.016				

Fig 4A–4F presented the surface response plots of various levels of particle size, solid: solvent ratio, time and temperature on diosgenin yield. The impact of extraction temperature and solid: solvent ratio on diosgenin extraction is given in (Fig 4A). At extraction temperature 45°C and solid: solvent ratio 1:45 g/ml, maximum diosgenin (1.204%) was attained. This shows that diosgenin yield was strongly influenced by these two parameters. (Fig 4B) shows that maximum diosgenin was extracted when temperature was 45°C and particle size 1.25 mm. (Fig 4C) indicates the evolution of diosgenin yield in accordance to time and extraction temperature. (Fig 4D) indicated that the maximum diosgenin was extracted at extraction time 45 min and particle size 1.25 mm. Increase in particle size causes decline in extraction of diosgenin. The effect of solid: solvent ratio and extraction time on the extraction diosgenin is shown in (Fig 4E). Maximum diosgenin was obtained at the solid: solvent ratio 1:45 and extraction time of 45 min. Effect of particle size and solid: solvent ratio on diosgenin extraction was shown in (Fig 4F). Particle size 1.25 mm and solid: solvent ratio of 1:45 (g/ml) shows maximum yield of diosgenin. Further, increase in both the parameters leads to decrease in the yield of diosgenin.

The article "Optimization of diosgenin extraction from Dioscorea deltoidea tubers using response surface methodology and artificial neural network modelling" was retracted in 2023. Reasons: errors in the images; duplicated images; overlap with earlier publications; a conflict of interest.

**Fig 4:** A. Three-dimensional surface response plots for diosgenin extraction at varying level of temperature and solid/solvent ratio. B. Contour plot for diosgenin extraction at varying level of temperature and particle size. C. Contour plot for diosgenin extraction at varying level of temperature and time. D. Contour plot for diosgenin extraction at varying level of time and particle size. E. Contour plot for diosgenin extraction at varying level of time and solid/solvent ratio. F. Contour plot for diosgenin extraction at varying level of particle size and solid/solvent ratio.

### 3.3 ANN modelling

In the present study, ANN adopted back propagation algorithm during training phase and was developed into 3 layers: input layer (X_2_, X_3_, X_4_, X_5_), hidden layer and output layer (% yield of diosgenin). In ANN modelling, 27 runs of BBD matrix were divided into 3 subsets, with approximate 19:4:4ratios to train, validate and test. The experimental data versus the computed ANN data in training, testing and validation networks is shown in Fig 5. The performance data obtained over entire training data and fitted at best epochs for validation data being represented (Fig 6). Similarly, gradient loss and training state achieved over entire ANN training is explained with the help of Fig 6. Best validation performance for the optimization of diosgenin was observed at epoch 15. The experimental results used for RSM was also applied to predict the optimal design of ANN (Table 9). In the experimental design, the selecting of appropriate numbers of neurons in the input, hidden and output layers were limited. In hidden layer number of neurons was selected when lowest error of predictive models attained. Initially, the neural network was optimized to acquire an ANN model with least dimension and errors in testing and training. The data apportioning (training, testing and validation) were accomplished to evade extreme training and over-parameterization. The goodness of fit between the observed and predicted response data form ANN models are shown in Fig 5 with correlation coefficients of 0.998% for extraction yield. Higher correlation coefficients reveal the reliability of the predictive models by ANN. For valid evaluation of predictive capability, a new validation data set (not belonging to the training data set previously used for model creation) of 9 runs was employed (Table 10).

The article "Optimization of diosgenin extraction from Dioscorea deltoidea tubers using response surface methodology and artificial neural network modelling" was retracted in 2023. Reasons: errors in the images; duplicated images; overlap with earlier publications; a conflict of interest.

**Fig 5:** Correlation between experimental versus computed yield of ANN.

**Fig 6:** A-B Performance data obtained (ANN) over entire training data and gradient loss for diosgenin.

**Table 9:** Comparison of predictive capacity of RSM and ANN models.

	RSM	ANN
Coefficient of determination(R^2^)	0.996	0.998
Root mean square error (RMSE)	0.001	0.001
Absolute average deviation (AAD)	0.018	0.018

**Table 10:** Validation data set for extraction variables with corresponding experimental and predicted value (RSM and ANN).

Run order	Factors				Diosgenin (% dry weight)		
	Solid: solvent ratio (X_2_)	Particle size (X_3_)	Time (X_4_)	Temperature(X_5_)	Experimental	RSM Predicted	ANN
**1**	50	0.2	20	50	1.125	1.121	1.127
**2**	50	2.0	20	50	1.137	1.133	1.136
**3**	50	0.2	80	50	1.135	1.132	1.137
**4**	50	2.0	80	50	1.131	1.130	1.134
**5**	20	1.1	20	50	1.119	1.117	1.119
**6**	80	1.1	20	50	1.137	1.138	1.137
**7**	20	1.1	80	50	1.136	1.132	1.135
**8**	80	1.1	80	50	1.126	1.122	1.126
**9**	50	0.2	50	20	1.144	1.146	1.144

Moreover, RSM model was compared with the ANN model that represented the ANN model as more accurate method of interpolation, prediction, and validation. In contrast to the RSM, ANN model showed less deviation between the predicted and experimental values. Table 6 depicted the predicted values in response to the experimental values obtained for diosgenin. In addition, comparison was drawn between two models on the basis of three significant statistical parameters, *viz*. Root mean square error (RMSE), Absolute average deviation (AAD) and regression coefficient (*r*^*2*^).

RMSE and AAD were calculated on the basis of Eqs 5 and 6.

Comparative overview of analytical parameters with RSM and ANN models are presented in Table 9. Though both RSM and ANN models showed good result of prediction, but higher R^2^ value and lower RMSE and AAD value revealed that ANN model can efficiently predict responses with greater evaluation abilities in comparison to RSM. This enhanced precision of the ANN can be caused by its universal capability to estimate the non-linearity, however RSM is simply based on a quadratic polynomial. Moreover, ANN has the capacity to estimate multi-response in a single procedure, while in RSM it has to be run separately. ANN revealed best validation statistical parameters, hence can be used as an accurate method in the optimization approaches [46–48].

The article "Optimization of diosgenin extraction from Dioscorea deltoidea tubers using response surface methodology and artificial neural network modelling" was retracted in 2023. Reasons: errors in the images; duplicated images; overlap with earlier publications; a conflict of interest.

## 4. Discussion

The present study involves the use of RSM to optimize extraction conditions for maximum diosgenin yield from *Dioscorea deltoidea* by using HPTLC analysis. The ANN model was used to simulate the data for the experiments done through RSM and to compare the values obtained experimentally (by RSM) and predictively (using ANN). The diosgenin yield can be influenced significantly by extraction parameters i.e solid: solvent, time, particle size and temperature. Low temperature was not suitable for extraction of bioactive compounds from the plant matrix due to inability to release the bioactive compounds. As the temperature rises the diosgenin yield increased but further increase in temperature had no effect on the diosgenin yield due to maximum diosgenin extracted from the plant matrix. Pandey et al. (2018) have reported the enhanced yield of pentacyclic triterpenoids from *Swertia chirata* stem at mean particle size (3 mm), temperature (65°C), and methanol–ethyl acetate solvent composition (45%) [45]. Similar results were found in our studies as particle size-temperature interaction was found to be significant. Diosgenin yield was maximum at optimized particle size due increase in the contact area of sample particles which is responsible for the better leaching of solute to reach the surface. Furthermore, very small particles may lead to technical difficulties related to the permeability of the solid bed, during the mixing of the plant material with solvent. Increased solubility of anthocyanins in solvents was found in extraction from black currants, due to increased temperature and sample to solvent ratio due better penetration of solvent into the plant matrix [29, 30]. Optimum extraction time is suitable for better extraction yield of bioactive compounds as we got in diosgenin yield. Likewise, results were obtained in bioactive compound yield from various medicinal plants [38–40]. RSM and ANN were efficaciously applied for optimization of extraction parameters for the extraction of diosgenin from *D*. *deltoidea*. For the optimization of diosgenin, seven different parameters (time, solvent composition, temperature, particle size solid: solvent ratio, pH and extraction cycles/steps) were run through PBD conditions and only four parameters (particle size; solid: solvent ratio; time and temperature) indicated significant impact on diosgenin extraction. The presence of interactions among the factors were studied and the interaction among solid: solvent ratio and particle size; time and particle size; particle size and temperature; solid: solvent ratio and time; and solid: solvent ratio and temperature revealed significant effects on diosgenin extraction.

The article "Optimization of diosgenin extraction from Dioscorea deltoidea tubers using response surface methodology and artificial neural network modelling" was retracted in 2023. Reasons: errors in the images; duplicated images; overlap with earlier publications; a conflict of interest.

## 5. Conclusions

BBD was used for the optimization of extraction factors and best extraction factors for diosgenin extraction were particle size (1.25 mm), solid: solvent ratio (1:45 g/ml), extraction temperature (45°C), and extraction time (45 min). The maximum experimental yield of diosgenin (1.204% dry weight) was observed close to the predicted value (1.202% dry weight) on the basis of the chosen optimal extraction factors. The developed mathematical model fitted well with experimental data for diosgenin extraction. The performance estimation results proposed that ANN as a modelling method was far superior to RSM. The present work is the first ever investigation of optimization of diosgenin extraction from *D*. *deltoidea* tuber using RSM and ANN. Moreover, further studies are crucial to design other modelling approaches that would enhance the synthesis of valuable bioactive compounds.
